This article has been retracted.

# Extraction of Long Time-Series Vegetation Indices from Combined Multisource Satellite Imagery

**DOI:** 10.1155/2022/3901372

**Published:** 2022-05-30

**Authors:** Yu Liu, Wenqing Li, Li Li, Naiqun Zhang

**Affiliations:** ^1^College of Life Sciences and Agricultural Engineering, Nanyang Normal University, Nanyang 473061, Henan, China; ^2^School of Civil Engineering and Architecture, Baise University, Baise 533000, Guangxi, China; ^3^Modern Agricultural Science and Engineering Institute, Tongji University, Shanghai 200082, China

## Abstract

Extracting vegetation cover information by combining multisource satellite images can improve the time scale of vegetation cover monitoring, realize encrypted observation in short period, and shorten the regional vegetation remote sensing monitoring cycle. The NDVI and RVI datasets from 2007–2019 were extracted using 9 phases of multisource satellite images (Landsat TM/OLI, Sentinel-2 MSI, and GF-1 PMS) covering Xiaxi, Sichuan. Three typical validation sites representing higher vegetation cover in mountains and no vegetation cover in water bodies in the region, respectively, were selected to extract NDVI and RVI at the corresponding locations. Linear regression and Spearman correlation coefficient (*ρ*) analysis were used to verify the correlation between NDVI and RVI from multisource images. The results showed that the vegetation indices fluctuated smoothly in the time series within the validation sites, and the vegetation indices of multisource satellite images were good measures of long-term vegetation cover in the region; the vegetation indices of the same satellite images showed significant correlations (both *R*^2^ and *ρ* exceeded 0.8), and the vegetation indices of different satellite images (PSM and MSI, PSM and OLI) showed more significant correlations (both *R*^2^ and *ρ* exceeded 0.7); the smaller the difference between the original resolutions of satellite images, the more significant the correlation between the extracted NDVI and RVI.

## 1. Introduction

Vegetation cover is a comprehensive quantitative index indicating the ground cover status of vegetation communities. Meanwhile, vegetation cover is also an important geoenvironmental factor to control soil erosion, soil invasion, and soil desertification. The traditional vegetation cover survey is generally based on manual sampling and observation. Although the measurement accuracy of this method is high, it is difficult to achieve quasi-real-time dynamic monitoring for large-scale vegetation cover survey. Secondly, manual sampling observation cannot obtain historical vegetation cover data. With the development of remote sensing observation technology and the open access to multisource satellite images (e.g., Landsat, Sentinel-2, and Gaofen 1/2 satellites, etc.), the dynamic measurement of vegetation cover over large areas in quasi-real time provides strong support. Several studies have shown that the vegetation indices extracted from satellite images can be a good measure of surface vegetation cover and its spatial and temporal evolution characteristics. For example, the extraction of vegetation indices using Landsat TM/OLI images [1–5], SPOT satellite images [6–8], HDS-1/2 satellite images [9–11], and Sentinel-2 satellite images [12–14] has provided basic data support for the spatial and temporal evolution of vegetation cover in the study area.

At present, studies generally focus on single satellite images to extract vegetation indices, while there are fewer relevant studies on joint multisource satellite images to extract vegetation indices. The differences between satellite payload indicators (spatial resolution, revisit period, orbit and band information, etc.) make it difficult to combine multisource satellite images for long time-series vegetation cover observation. For example, there are large differences in spatial resolution, spectral range, and revisit period (30 m, 10 m, and 2 m, respectively) among Landsat-8, Sentinel-2, and HMS-1/2 satellite images, which make it difficult to unify the joint multisource satellite images on the scale. However, the significance of joint multisource satellite images to extract vegetation cover is (1) to realize the complementary advantages of multisource satellite images, so as to obtain high-resolution and higher-accuracy vegetation cover data; (2) to improve the time scale of satellite images for vegetation cover monitoring and realize long time series regional vegetation cover monitoring; (3) to provide dense satellite images in a short period and shorten the regional vegetation cover monitoring cycle. Therefore, this paper aims to explore the extraction of long time-series vegetation indices based on multisource satellite images (Landsat, Sentinel-2, and GF-1). Taking Xiaxi Township in Sichuan Province as an example, the feasibility of joint multisource satellite images to obtain long time series vegetation indices is discussed.

## 2. Data and Methods

The test area selected for this paper is Xiaxi Township, Pingshan County, Yibin City, Sichuan Province (hereinafter referred to as the test area). The administrative area of the test area is 70.98 km^2^, and the GF-1 fusion image (2m) and digital elevation model show that the middle water system of the area is developed with rivers and sufficient water supply, and the surrounding area is mainly mountainous with good vegetation cover (Figure 1). In addition, Landsat, Sentinel-2, and GF-1 satellite images all covered the area.

### 2.1. Remote Sensing Data

Landsat TM/OLI images were obtained from the Earth Resources Observation and Science Center (EROS) of the United States Geological Survey (USGS), with 6 image periods imaged in September 2007, June 2009, June 2011, May 2013, and October 2015 Sentinel-2 MSI images from ESA (European Space Agency, https://scihub.copernicus.eu), with 2 image phases imaged in September 2017 and June 2018. GF-1 PMS images are from the China Resources Satellite Center's Land Observation Satellite Data Service Platform, and the imaging time is June 2019. All satellite images (9 issues) covered the test area spatially and the plant growth period temporally, and the total cloudiness in the area was controlled below 5%.

### 2.2. Data Preprocessing

Due to the existence of complex feature information such as spatial spectra, radiometric resolution, and nonvegetation cover change signals caused by long time sequences among multisource satellite images, which will reduce the quality of regional vegetation cover information extraction to a certain extent. Therefore, before the extraction of vegetation cover information, preprocessing of multisource satellite images is needed to correct the geometric distortion and radiometric deformation between the original images, minimize the distortion, distortion, noise, blur, and spatial position deviation when imaging, and obtain relatively realistic images. Image preprocessing includes radiometric calibration (to reduce inter-annual image reflection differences), FLASSH atmospheric correction (to eliminate images reflected by atmospheric molecules and aerosol scattering, light, and other factors on features), geometric correction (to limit images from Earth curvature, satellite attitude, sensor position, etc.), orthorectification correction (tilt and projection aberration correction), image fusion (based on CN spectral sharpening-based multispectral and panchromatic band fusion), and image alignment (aligning and resampling other images with the GF-1 image as the primary image). Finally, a multisource satellite image dataset covering the test area for the long time series from 2007 to 2019 was obtained. The image preprocessing process is shown in Figure 2.

### 2.3. Vegetation Index

Vegetation Index (VI) refers to various values with certain intellectual significance to vegetation, which are formed by linear or nonlinear combination of multispectral information acquired by satellite sensors. The vegetation index is a characteristic index calculated based on the characteristics of vegetation reflection band to reflect the growth status, coverage, and vegetation volume of the ground. In this paper, two vegetation indices, NDVI and RVI [15], which are commonly used in remote sensing monitoring of vegetation cover, are selected to verify the feasibility of joint multisource satellite image long time-series vegetation cover observation.

(1) NDVI (normalized difference vegetation index) is calculated by
  (1) $$\begin{array}{c} \text{NDVI}=\frac{\rho_{\text{NIR}}-\rho_{R}}{\rho_{\text{NIR}}+\rho_{R}}. \end{array}$$
(2) RVI (ratio vegetation index) is calculated by
  (2) $$\begin{array}{c} \text{RVI}=\frac{\rho_{R}}{\rho_{\text{NIR}}}, \end{array}$$
where and denote the near-infrared band and infrared band feature reflectance, respectively.

## 3. Results and Analysis

### 3.1. Vegetation Index Calculation Results

In this paper, the normalized vegetation index (NDVI; Figure 3) and ratio index (RVI; Figure 4) datasets were extracted corresponding from the 9-period normalized vegetation index (NDVI; Figure 3) and ratio index (RVI; Figure 4) datasets in the test area from 2007–2019 using preprocessed multisource satellite image datasets (GF-1 PMS images, Sentinel-2 MSI images, and Landsat TM/OLI images). Three representative validation sites were selected in the test area, representing typical higher vegetation cover in mountainous areas (R1 and R3) and no vegetation cover within water systems (R2). The results showed that the NDVI values of R2 were all less than 0, which was consistent with the relationship that negative NDVI values indicated that the ground cover was nonvegetation cover such as water system (Figure 5); the NDVI values extracted at R1 and R3 were both above 0.5, indicating that both of them were vegetation cover areas, which was consistent with the mountain vegetation cover shown by the fused GF-1 image in Figure 5. The comparison results of RVI in typical areas show that the RVI values at R2 are basically close to 1 (the ground cover corresponding to RVI near 1 is artificial buildings, water systems, etc.); the RVI values at R1 and R3 are both above 4.0, which is consistent with the qualitative analysis rule that the RVI of green and healthy vegetation cover areas is much larger than 1 [16].

In addition, although the 9-period NDVI and RVI extracted from four types of satellite images (Landsat TM, Landsat OLI, Sentinel-2 MSI, and GF-1PMS images) cover 12 years (2007–2019) in time scale. However, the NDVI and RVI values within the typical area fluctuated smoothly in the time series, which reasonably reflects the pattern of ground vegetation cover distribution during the growing season in a relatively stable geographic environment. This also indicates that the vegetation index by combining multisource satellite images is still a good measure of the long-term vegetation cover status. Therefore, based on the typical regional statistical results and the spatial distribution of NDVI and RVI of the four types of satellite images in the test area, there is a strong correlation between the long-term serial vegetation cover and the vegetation indices extracted from the multisource satellite images in the test area [17].

### 3.2. Correlation Analysis of Vegetation Indices

In order to verify the correlation and stability between the vegetation indices extracted using multisource satellite images, a one-dimensional linear regression analysis was performed between the vegetation indices calculated from the same satellite and different satellite images. Theoretically, the higher the slope K and the higher the correlation coefficient *R* of the linear regression relationship, the higher the correlation between the two indices. Meanwhile, Spearman's correlation coefficient was introduced as a measure of the correlation between the two vegetation indices for the following reasons: (1) Spearman's correlation coefficient is a rank correlation coefficient, which estimates the position of the variables within the overall data for correlation calculation. Because of the positive correlation that the larger the vegetation index value (NDVI > 0) is, the larger the ground vegetation cover is, the introduction of Spearman's correlation coefficient can better measure the correlation between vegetation indices; (2) Spearman's correlation coefficient has no limitation on whether the data conform to normal distribution and the sample size. The formula for calculating Spearman's correlation coefficient (*ρ*) is as follows:

(3) $$\begin{array}{c} \rho =\frac{\sum_{i}\left(x_{i}-\bar{x}\right)\left(y_{i}-\bar{y}\right)}{\sqrt{\sum_{i}{\left(x_{i}-\bar{x}\right)}^{2}\sum_{i}{\left(y_{i}-\bar{y}\right)}^{2}}}. \end{array}$$

The correlation analysis of NDVI of the four types of images produced eight linear regression equations and corresponding Spearman correlation coefficients to represent the correlation between NDVI of the same satellite and different satellite satellite images, respectively. Specifically, between Landsat TM images, between Landsat OLI images, between Landsat TM and Landsat OLI images, between Sentinel MSI images, between GF-1 PSM and Sentinel MSI images, between GF-1 PSM and Landsat OLI images, between Landsat OLI and Sentinel MSI images, and the correlation between GF-1 PSM and Landsat TM images. The linear regression equations all passed the significance test (*p* > 0.05) and were statistically significant, and the coefficient of determination *R*^2^ and Spearman correlation coefficient *ρ* were both higher than 0.6. This indicates that all four types of image NDVI showed significant correlation between NDVI at the confidence level of 0.05. By longitudinal comparison, it can be seen that the determination coefficients *R*^2^ between Landsat TM, Landsat OLI, and Sentinel MSI images with different imaging times reach 0.8043, 0.8513, and 0.8383, respectively (Table 1), indicating the best correlation between NDVI of the same satellite images. Secondly, the correlations between GF-1 PSM and Sentinel MSI image NDVI and GF-1 PSM and Landsat OLI image NDVI are also significant (the corresponding *R*^2^ and Spearman's correlation coefficients are over 0.7), which represent the strong correlation between NDVI of different satellite images in different time phases. This also indicates that different satellite images of different phases can be used jointly for vegetation cover monitoring in the same area, thus extending the temporal coverage of regional vegetation cover status and achieving encrypted observation in short time period to a certain extent and obtaining quasi-real-time vegetation cover observation results with longer time series or shorter revisit period than that of a single satellite. As shown in Table 2 that the determination coefficient *R*^2^ and correlation coefficient *ρ* between Landsat TM and Landsat OLI image NDVI, Landsat OLI and Sentinel MSI image NDVI, and GF-1 PMS and Landsat TM image NDVI are basically lower than 0.7, indicating that the correlation between these three images NDVI is low. This low correlation will make the uncertainty of NDVI results increase throughout the monitoring cycle and introduce bias to further constrain the vegetation cover.

## 4. Conclusions

The NDVI and RVI datasets for 2007–2019 were extracted using 9-phase multisource satellite images (Landsat TM/OLI, Sentinel-2 MSI, and GF-1 PMS) covering the experimental area. Three typical validation sites representing higher vegetation cover in mountains (R1 and R3) and no vegetation cover in water bodies (R2) in the region were selected to extract NDVI and RVI at the corresponding locations. Linear regression and Spearman correlation coefficient (*ρ*) analysis were used to verify the correlation between NDVI and RVI from multisource satellite images. The results show that the NDVI and RVI extracted from the validation sites can well distinguish vegetation cover from nonvegetation cover, and the two vegetation indices fluctuate smoothly along the time series, and the vegetation indices of multisource satellite images can well measure the long-term vegetation cover in the region; the vegetation indices of the same satellite images show significant correlation (*R*^2^ and *ρ* exceed 0.8), and the vegetation indices between different satellite images (GF-1 PSM and Sentinel MSI, GF-1 PSM, and Landsat OLI) showed significant correlation (*R*^2^ and *ρ* exceeded 0.7), while the correlation between vegetation indices of other different images was low; through horizontal and vertical comparison of correlation coefficients.

## Figures and Tables

**Figure 1:** GF-1 fusion image and digital elevation model of the test area. GF-1 fusion image: color composite 3, 2, 1 band (RGB); digital elevation model (DEM) from the SRTM (Shuttle Radar Topography Mission) 30m DEM published by NASA. (a) Regional GF-1 fusion image (2 m). (b) Regional Digital Elevation Model.

**Figure 2:** Multisource satellite image preprocessing process and method. FLAASH: atmospheric correction model (fast line-of-sight atmospheric analysis of spectral hypercubes). Sen2Cor: processor generated by Sentinel-2 class 2A products, which automatically performs radiometric calibration, atmospheric correction, cirrus processing, etc.

**Figure 3:** NDVI results of multisource satellite imagery in the test area from 2007–2019. Landsat NDVI: NDVI extracted using 6-phase fusion-aligned Landsat TM/OLI imagery; Sentinel-2 NDVI: NDVI extracted using 2-phase fusion-aligned Sentinel-2 MSI imagery; GF-1 NDVI: NDVI extracted using fused GF-1 PMS imagery. Black (R2) and purple (R3) indicate the NDVI comparison analysis positions, respectively.

**Figure 4:** RVI results of multisource satellite imagery in the test area from 2007–2019. Landsat RVI: RVI extracted using 6-phase fusion-aligned Landsat TM/OLI imagery; Sentinel-2 RVI: RVI extracted using 2-phase fusion-aligned Sentinel-2 MSI imagery; GF-1 RVI: RVI extracted using fused GF-1 PMS imagery. Blue (R1), black (R2), and purple (R3) indicate RVI contrast analysis positions, respectively.

**Figure 5:** Time series NDVI and RVI extraction results within a typical region. R1, R2 and R3 denote the NDVI and RVI values within a typical region of the selected area, respectively, and the corresponding positions are shown in Figures 3 and 4.

**Table 1:** NDVI correlation analysis of Landsat TM/OLI, Sentinel-2 MSI, and GF-1 PMS images.

Data types	Data types	Slope K (95% confidence interval)	Intercept (95% confidence interval)	Linear regression equations	Decision factor *R*^2^	Correlation coefficient *ρ*
2007 TM	2009 TM	0.7769 (0.7458, 0.808)	0.1589 (0.1395, 0.1783)	*y* = 0.7769*x* + 0.1589	0.8043	0.8453
2013 OLI	2015 OLI	0.3704 (0.354, 0.3868)	0.5149 (0.505, 0.5248)	*y* = 0.3704*x* + 0.5149	0.8513	0.8751
2009 TM	2013 OLI	0.7769 (0.7458, 0.808)	0.1589 (0.1395, 0.1783)	*y* = 0.7769*x* + 0.1589	0.6817	0.7037
2017 MSI	2018 MSI	0.7667 (0.7266, 0.7969)	−0.0878 (−0.1048, −0.0708)	*y* = 0.7667*x* − 0.0878	0.8383	0.8869
2019 PSM	2018 MSI	0.6909 (0.6615, 0.7204)	0.1324 (0.1167, 0.1482)	*y* = 0.6909*x* + 0.1324	0.7858	0.8063
2019 PSM	2019 OLI	0.6729 (0.6305, 0.7153)	0.2286 (0.2058, 0.2514)	*y* = 0.6729*x* + 0.2286	0.7043	0.7343
2019 OLI	2018 MSI	0.4251 (0.4012, 0.449)	0.5375 (0.5265, 0.5484)	*y* = 0.4251*x* + 0.5375	0.6737	0.6924
2019 PSM	2011 TM	0.9235 (0.8682, 0.9788)	−0.0735 (−0.1131, −0.03391)	*y* = 0.9235*x* − 0.0735	0.6031	0.6375

**Table 2:** Correlation analysis of Landsat TM/OLI, Sentinel-2 MSI, and GF-1 PMS image RVI.

Data types	Data types	Slope K (95% confidence interval)	Intercept (95% confidence interval)	Linear regression equations	Decision factor, *R*^2^	Correlation coefficient, *ρ*
2007 TM	2009 TM	0.8943 (0.8569, 0.9317)	0.954 (0.7856, 1.122)	*y* = 0.8943*x* + 0.954	0.8132	0.8382
2013 OLI	2015 OLI	1.094 (1.058, 1.131)	2.57 (2.409, 2.73)	*y* = 1.094*x* + 2.57	0.8252	0.8597
2009 TM	2013 OLI	0.5754 (0.5498, 0.601)	1.34 (1.209, 1.47)	*y* = 0.5754*x* + 1.34	0.6655	0.6949
2017 MSI	2018 MSI	0.8257 (0.8117, 0.8396)	1.67 (1.633, 1.707)	*y* = 0.8257*x* + 1.367	0.9136	0.9537
2019 PSM	2018 MSI	0.6724 (0.6432, 0.7015)	1.789 (1.707, 1.87)	*y* = 0.6724*x* + 1.789	0.8159	0.8511
2019 PSM	2019 OLI	1.111 (1.02, 1.202)	1.404 (1.093, 1.716)	*y* = 1.111*x* + 1.404	0.7637	0.7870
2019 OLI	2018 MSI	0.6738 (0.6601, 0.6875)	3.452 (3.306, 3.597)	*y* = 0.6738*x* + 3.452	0.7059	0.7212
2019 PSM	2011 TM	0.8424 (0.7919, 0.8928)	2.08 (1.908, 2.253)	*y* = 0.8424*x* + 1.34	0.6351	0.6513

## Data Availability

The raw data supporting the conclusions of this article will be made available by the authors, without undue reservation.
